# Clinical Observation of Zhengyuan Capsule Combined with Neoadjuvant Chemotherapy for Triple-Negative Breast Cancer

**DOI:** 10.1155/2022/1375724

**Published:** 2022-05-23

**Authors:** Xiaoyu Zhang, Huixin Li, Feng Wu, Dan Sun, Hengle Zhang, Lijun Jin, Xiaoning Kang, Zunyi Wang

**Affiliations:** ^1^Cangzhou Central Hospital, Cangzhou, China; ^2^Hebei Medical University, Cangzhou Central Hospital Affiliated to Hebei Medical University, Cangzhou, China

## Abstract

**Objective:**

To study the clinical effect of Zhengyuan capsule combined with neoadjuvant chemotherapy in the treatment of triple-negative breast cancer (TNBC).

**Methods:**

From September 2014 to September 2017, 120 TNBC patients who underwent radical mastectomy in our hospital were randomly divided into control group (*n* = 60) and observation group (*n* = 60). The short-term curative effect, the incidence of toxicity and side effects, and the score of quality of life of the patients were compared. Both recurrence and metastasis rates were also analyzed.

**Results:**

The combined treatment of Zhengyuan capsule with neoadjuvant chemotherapy significantly improved the objective remission rate (70.00% in the observation group versus 40.00% in the control group) (*P* < 0.05). Moreover, this combined treatment significantly decreased the total incidence of side effects (35.00% versus 75.00%). Accordingly, the score of quality of life was also increased in patients treated with Zhengyuan capsule plus neoadjuvant chemotherapy (*P* < 0.05). Furthermore, supplementation of Zhengyuan capsule can significantly suppress both the recurrence and metastasis rate of TNBC in patients treated with neoadjuvant chemotherapy after radical mastectomy in following 3 years (30.00% versus 10.00%, *P* < 0.05).

**Conclusion:**

Zhengyuan capsule effectively improves the short-term curative effect, reduces the side effects of chemotherapy, and improves the quality of life of patients treated with neoadjuvant chemotherapy after radical mastectomy. More importantly, this combined treatment can also reduce the long-term recurrence and metastasis of TNBC.

## 1. Introduction

As a special type of breast cancer, triple-negative breast cancer (TNBC) exhibits malignant phonotypes and develops rapidly, which has high rate of recurrence and metastasis in the long term after radical mastectomy, eventually resulting in poor outcome [1]. In recent years, clinical studies have found that neoadjuvant chemotherapy (NAC) is an effective treatment for patients with locally advanced breast cancer. NAC can effectively reduce the tumor size to increase the success rate of surgical resection and breast-conserving surgery, but it has great side effects on patients with cancer [2]. Zhengyuan capsule is composed of masturbation sheep bud, Huang Geng, raw sun ginseng, *Atractylodes macrocephala*, tortoise plate, whole nail, privet seed, tangerine peel, and so on. It has the function of tonifying qi, invigorating kidney, and dispersing blood stasis and aims at the pathogenesis treatment of cancer [3]. At present, there are few reports on the combination of Zhengyuan capsule and neoadjuvant chemotherapy in China. The purpose of this study was to explore the clinical effect of Zhengyuan capsule combined with neoadjuvant chemotherapy in the treatment of TNBC.

## 2. Materials and Methods

### 2.1. General Information

A total of 120 patients with TNBC who underwent radical mastectomy in our hospital from September 2014 to September 2017 were selected. According to the computer random number grouping method, 120 patients with TNBC were randomly divided into control group (*n* = 60) and observation group (*n* = 60). The general clinical data of the two groups were compared (*P* > 0.05). The data are as follows. The age of the control group was with an average age of (53.85 ± 10.35) years, including 54 cases of invasive ductal carcinoma and 6 cases of invasive lobular carcinoma, while that of the observation group was with an average age of (55.50 ± 8.63) years old, including 51 cases of invasive ductal carcinoma and 9 cases of invasive lobular carcinoma. This study was approved by the Ethics Committee (approval no. 2013-187-20). All patients provided the signed informed consent.

### 2.2. Inclusion Criteria

- All selected patients met the diagnostic criteria of breast cancer in the guidelines and norms for diagnosis and treatment of breast cancer of China Anti-Cancer Association (2008 Edition) and then diagnosed as stage IIb and III by pathology
- Biopsies were performed by Memeton or hollow needle before NAC implementation
- Complete pathological results and lymph node metastasis were obtained

### 2.3. Exclusion Criteria

- Cancer tissues with positive expression of HER-2 and/or HR
- Patients with severe organ dysfunction such as the heart, liver, kidney, acute, or chronic infectious diseases
- Pregnant or lactating women
- Metastatic breast cancer or distant metastasis
- Allergic constitution, with contraindications to research drugs
- Those whose expected survival time of less than 3 months
- Patients with incomplete clinical data or unwilling to sign informed consent form

### 2.4. Methods

The control group was given neoadjuvant chemotherapy after operation, and cyclophosphamide 600 mg/m^2^ plus doxorubicin 60 mg/m^2^ plus docetaxel 100 mg/m^2^ regimen was selected. The drug was given on the first day, intravenous drip, for 3 weeks as a course of treatment for 6 consecutive courses. The observation group was treated with Zhengyuan capsule on the basis of the control group, and the chemotherapy scheme was the same as that of the control group. Zhengyuan capsule was treated with Zhengyuan capsule (Yangzijiang Pharmaceutical Group Guangzhou Hairui Pharmaceutical Co., Ltd., Z20148001). The dosage of Zhengyuan capsule was taken orally in remission period, 3 times a day, for 8 weeks.

### 2.5. Observation Indices

The short-term efficacy, the incidence of toxicity and side effects, and the score of quality of life of the patients with triple-negative breast cancer were compared between the two groups. The quality of life was evaluated using Generic Quality of Life Inventory-74 (GQOL-74) that comprises four dimensions: physical health, mental health, social function, and material life. The score of a single dimension was 100. The higher the score, the better the quality of life of this dimension, and the follow-up observation for 3 years. The recurrence and metastasis rates of the two groups were compared.

### 2.6. Curative Effect Evaluation

The evaluation of curative effect can be divided according to the situation of tumor focus and the occurrence of side effects as follows: complete remission (CR): lesions basically disappeared, and no side effects occurred; partial remission (PR): lesions decreased by more than 30%, and the side effects were not obvious; stable (SD): lesions decreased by less than 30% or enlarged by less than 20%, and the toxicity and side effects were not obvious. The enlarged range of lesions in progressive (PD) was more than 20%, and the toxic and side effects were serious. Objective remission rate = CR + PR.

### 2.7. Statistical Analysis

SPSS 22.0 software was used to process the data, *χ*^2^ test was used to compare the counting data, and *t*-test was used to compare the measurement data, which showed (case, %) and mean ± standard deviation, *P* < 0.05, that is, statistically significant.

## 3. Results

### 3.1. General Analysis of Clinical Features of Patients between the Two Groups

As shown in Table 1, no significant difference was in general clinical data such as age, pathological classification, and TNM stage between the two groups (*P* > 0.05).

### 3.2. Comparison of Short-Term Efficacy in Presence or Absence of Zhengyuan Capsule

As shown in Table 2, the treatment of Zhengyuan capsule significantly improved the objective remission rate (ORR) as relative to those in the control group (70.00% versus 40.00%), which indicated that supplementation of Zhengyuan capsule enhanced the tumor-suppressive effects of neoadjuvant chemotherapy.

### 3.3. Comparison of the Incidence of Side Effects of Neoadjuvant Chemotherapy

In addition to the tumor-suppressive effects, neoadjuvant chemotherapy also elicited toxic to patient's health. To investigate the role of Zhengyuan capsule on the side effects of neoadjuvant chemotherapy, we analyzed the total incidence of side effects between the two groups. As shown in Table 3, administration of Zhengyuan capsule significantly attenuated the side effects of chemotherapy (35% versus 75%, *P* < 0.05).

### 3.4. Comparison of Living Quality of Patients with TNBC

We next focused on the effects of Zhengyuan capsule on improvement of the quality of life. As shown in Table 4, compared with the control group, the score of quality of life in the observation group was higher than those in the control group (*P* < 0.05), suggesting the positive role of Zhengyuan capsule on improvement of the quality of life.

### 3.5. Comparison of Long-Term Recurrence and Metastasis Rates between the Two Groups

After follow-up for 3 years, compared to 18 cases of recurrence and metastasis in the control group, with a recurrence and metastasis rate of 30.00%, 6 cases of recurrence and metastasis were observed in the observation group, with a recurrence and metastasis rate of 10.00%. Statistical analysis revealed that the treatment of Zhengyuan capsule elicits suppressive effects on the recurrence and metastasis of TNBC (*P* < 0.05).

## 4. Discussion

Triple-negative breast cancer (TNBC) is defined as breast cancer in which estrogen receptor (ER), progesterone receptor (PR), and human epidermal growth factor receptor 2 (HER-2) are all negative [4]. In recent years, the incidence of TNBC is increasing, and its proportion in breast cancer is also gradually increasing. Distinct from other breast cancer, the incidence of triple-negative breast cancer in young women is also higher, coupled with the larger size of the tumor. Relatively, TNBC develops rapidly and its outcome and morbidity within 5 years are poor and very high, respectively [5].

To date, the pathogenesis of TNBC is not clear. Due to lack of specific treatment, radical mastectomy is often employed for the treatment of TNBC. Moreover, the patients are prone to recurrence and metastasis after operation, and the prognosis is relatively disadvantageous [6–8]. It is reported that neoadjuvant chemotherapy exhibits suppressive effects on the lesions of triple-negative breast cancer after operation [9]. However, postoperative chemotherapy is not effective in the prevention of long-term recurrence and metastasis in patients with TNBC, and the side effects of radical mastectomy are also toxic to patients.

In recent years, traditional Chinese medicine has been gradually used in the treatment of TNBC. Traditional Chinese medicine believes that in the process of clinical antitumor treatment, radiotherapy, and chemotherapy, targeted therapy, immunotherapy, and other therapeutic measures or factors can damage the vital energy of the human body, coupled with tumor consumption. Deficiency of vital qi for a long while in turn results in fatigue, insomnia, emotional loss, and other symptoms of fatigue. Zhengyuan capsule is composed of epimedium, astragalus, raw ginseng, Atractylodes macrocephala, tortoise plate, turtle shell, privet seed, tangerine peel, and so on. In the prescription, epimedium is warm, tasty, and sweet, returning to the liver and kidney meridians, warming the kidney and strengthening yang, and tonifying the liver and kidney, for the king's medicine [10]. Astragalus helps to invigorate the spleen and qi, elevate Yang depression, invigorate the lungs, and enhance immunity; washing raw ginseng and drying it can help to invigorate vitality, invigorate the spleen and lung, and nourish the tendons and soothe the nerves; Atractylodes can help invigorate the spleen. Invigorating Qi and promoting blood circulation, resolving phlegm and phlegm, and combining the above several types as the research object, it has the functions of invigorating the spleen and lung, invigorating qi and promoting blood circulation, invigorating the spleen and resolving phlegm. Turtle plate nourishes yin and yang, nourishes kidney and bones, nourishes blood, and nourishes heart. Tortoise shell nourishes yin and nourishes yang, disperses knots, and is soft and firm. Ligustrum lucidum nourishes liver and kidney yin and improves eyesight. The three are combined as adjuvant drugs, which can tonify the yin of the liver and kidney, nourish yin and nourish blood, and soften and disperse knots, and the medicinal properties are cold and cool, making the whole prescription warm but not dry [11]. Then, we used tangerine peel as the medicine, which is warm in nature with bitter taste, for spleen and lung meridian, regulating qi and resolving phlegm to disperse the knot, so that the whole prescription will be loose, tonic but not stagnant, and will not be too greasy. The above eight drugs combined with warm but not dry, nourishing but not greasy, together play the function of tonifying qi and invigorating spleen, tonifying kidney and filling essence, regulating qi and resolving phlegm, and softening and dispersing knots, which can be used in the treatment of cancer-related fatigue [12, 13]. In the previous study, Guan [14] and others confirmed that Zhengyuan capsule played a role mainly by increasing the amount of liver glycogen and enhancing hematopoiesis and immune function, but also through the effect on thyroid function.

Here, we found that the combined treatment of Zhengyuan capsule with neoadjuvant chemotherapy significantly improved the objective remission rate and the quality of life (*P* < 0.05). The total incidence of side effects in the observation group was lower than that in the control group (*P* < 0.05). The long-term recurrence and metastasis rate in the control group was also lower than that in the control group (*P* < 0.05); it fully shows that Zhengyuan capsule has a significant therapeutic effect on the treatment of TNBC, which can effectively control the tumor progress and reduce the long-term recurrence and metastasis, mainly because these two kinds of traditional Chinese medicine are used in combination with neoadjuvant chemotherapy. It can reduce the side effects caused by chemotherapy, which in turn ensures that the treatment can be carried out smoothly.

To sum up, during the period of neoadjuvant chemotherapy after radical mastectomy, Zhengyuan capsule can effectively improve the short-term efficacy of patients, reduce the side effects of chemotherapy, and improve their quality of life. More importantly, the combinational treatment of Zhengyuan capsule with neoadjuvant chemotherapy can reduce the long-term recurrence and metastasis of TNBC.

## Figures and Tables

**Table 1:** Comparison of clinical data of patients with TNBC.

Group	Case	Average age	Lymphatic	Bone	Liver	Lung	Soft tissue	TNM stage (years)	
								IIb	III
Observation	60	55.50 ± 8.63	36	39	24	33	30	24	36
Control	60	53.85 ± 10.35	39	33	30	27	42	21	39

**Table 2:** Comparison of short-term efficacy of TNBC (case, %).

Group	Case	CR	PR	Stability	Progression	ORR
Observation	60	15 (25.00)	27 (45.00)	15 (25.00)	3 (5.00)	42 (70.00)
Control	60	6 (10.00)	15 (25.00)	27 (45.00)	12 (20.00)	24 (40.00)
*X* ^2^						10.909
*P* value						0.001

*Note.* CR: complete remission; PR: partial remission; ORR: objective remission rate.

**Table 3:** Comparison of the incidence of side effects of TNBC (case, %).

Group	Case	MS	GR	SKP	Headache	Incidence
Observation	60	6 (10.00)	9 (15.00)	3 (5.00)	3 (5.00)	21 (35.00)
Control	60	9 (15.00)	15 (25.00)	12 (20.00)	9 (15.00)	45 (75.00)
*X* ^2^						19.394
*P* value						≤0.001

*Note.* MS: myelosuppression; GR: gastrointestinal reaction; SKP: skeletal muscle pain.

**Table 4:** Comparison of quality of life scores of patients with TNBC (mean ± standard deviation).

Group	Case	Physical health	Psychological health	Social health	Material living
Observation	60	81.85 ± 3.03	82.00 ± 3.19	81.56 ± 2.82	82.36 ± 2.63
Control	60	70.80 ± 2.49	72.78 ± 2.45	70.05 ± 2.38	70.57 ± 2.50
*t*		21.841	17.723	24.156	25.171
*P* value		≤0.001	≤0.001	≤0.001	≤0.001

## Data Availability

The datasets used during the present study are available from the corresponding author upon reasonable request.
